The article "Does industrial up-gradation, environment regulations, and resource allocation impact on foreign direct investment: Empirical evidence from China" was retracted in 2025. Reasons: an official misconduct investigation; compromised peer review; a compromised editor; unreliable results or conclusions.

# Does industrial up-gradation, environment regulations, and resource allocation impact on foreign direct investment: Empirical evidence from China

**DOI:** 10.3389/fpsyg.2022.999953

**Published:** 2022-10-24

**Authors:** Jiacai Xiong, Linghong Chen

**Affiliations:** School of Accounting, Jiangxi University of Finance and Economics, Nanchang, China

**Keywords:** industrial upgradation, environmental regulations, resource allocation, FDI inflows, China

## Abstract

Because of China’s tremendous increase in foreign direct investment (FDI) over the past two decades, this method of internationalization has become increasingly significant for companies worldwide. Heavy industry’s dominant role in China’s industrial structure must be modernized to ensure the country’s long-term growth and prosperity. There are 30 provinces in China covered by this dataset, which dates back from 2005 to 2018. Augmented mean group (AMG) and common correlated effects mean groups (CCE-MG) estimations demonstrate that China’s industrial upgrading and resource allocation considerably impact FDI inflows. The findings show that FDI inflows appear to be negatively affected by environmental rules. The results show that industrial upgradation and environmental regulations have not had the expected effect on FDI in China without the participation of other stakeholders. For the selected panel, the results from the control variable show that population aging reduces foreign direct investment inflows, whereas, economic growth increases FDI inflows. According to our findings and those of the empirical study, we make some policy proposals to help Chinese provinces attract more foreign direct investment by encouraging and upgrading the screening of such investments.

## Introduction

As the global economy has become more interconnected, so has the volume of FDI. Countries worldwide are tightening environmental regulations in response to the deterioration of the global environment (Taiwo Onifade et al., 2021); this is becoming a significant issue that influences organizations’ investment decisions and financial performance (Dong et al., 2021). As a result of globalization, firms can spread their manufacturing processes to other parts of the world, making environmental regulations less strict and a possible source of relative advantage in FDI (Erdoğan et al., 2022). There have been significant efforts by policymakers to attract FDI recently, and Abdur et al. (2022) have highlighted the contributing factors critical for investment decisions. A lot of research focuses on the importance of infrastructure and market size in attracting foreign investment (FDI) (Gao et al., 2020; Chen et al., 2021; Lei et al., 2021). In the long history of attracting FDI, China has been a prominent actor and continues to be so (Zhang et al., 2021a). The capacity for technical innovation has grown recently as FDI has risen (Dong et al., 2021). Several environmental legislation has lately been developed to deal with external and local pressure to improve environmental quality (Qin, 2021). Outward FDI in China has seen a significant shift in 2013 due to the BRI-Belt and Road Initiative’s promotion, focusing on the economic integration of regions at the industrial level across countries (Pavlichenko et al., 2021; Onifade et al., 2022a).

The article "Does industrial up-gradation, environment regulations, and resource allocation impact on foreign direct investment: Empirical evidence from China" was retracted in 2025. Reasons: an official misconduct investigation; compromised peer review; a compromised editor; unreliable results or conclusions.

Due to the rapid rise of China’s industrial sector during the 1980s, most Chinese cities have seen tremendous growth in their economies (Sokhanvar, 2019). Given that the heavy industry sector is the primary consumer and emits air pollutants, an imbalanced industrial structure with a very high proportionality of the industrial sector would result in substantial resource misallocation, serious environmental pollution, and even massive health losses, which greatly hindered the sustainable development of China (Alola and Onifade, 2022; Onifade et al., 2022b). There have been a lot of efforts in recent years by the Chinese government to improve their economy, such as developing seven important rising industries in 2010 and creating a 2025 plan called Made in China 2025 (Zhao et al., 2021a,b; Xu et al., 2022; Zhou et al., 2022a). Furthermore, it is advocated that the modern service industry be integrated with the sophisticated manufacturing industry. Numerous studies examine the factors that influence the modernization of the industrial structure at the national and regional levels. Studies focusing on international trade, which substantially impacts local competition, foreign capital inflows, and export growth, are prevalent in the literature (Ai et al., 2021). Local enterprises frequently drive efforts to upgrade the industrial base, but the degree of human capital, technical assistance, financial development, and institutional quality also plays a significant role in this process (Hu F. et al., 2021; Song et al., 2021; Zhou et al., 2022b). As the environment has deteriorated to an alarming degree, an increasing number of academics have focused on the impact of environmental legislation on the industry’s structure (He et al., 2020). When economic incentives influence municipal governments, the ineffective implementation of environmental regulations is a major roadblock to attaining the aim (Wang and Wang, 2021). Environmental information available to the public could help address non-compliance issues like these and refill the current environmental governance system simultaneously.

The article "Does industrial up-gradation, environment regulations, and resource allocation impact on foreign direct investment: Empirical evidence from China" was retracted in 2025. Reasons: an official misconduct investigation; compromised peer review; a compromised editor; unreliable results or conclusions.

Upgrading the regional industrial structure includes transitioning from primary and secondary industries to tertiary industries, represented in the distribution of production value among various regional sectors (Bashir et al., 2021). Environmental rules can be tightened through the ecological information disclosure program, which could improve the industrial structure. Companies in more transparent cities are subject to stricter regulations because of their ability to handle rebellious local governments and pollutants successfully. Environmental regulation’s increased compliance costs may drive polluting companies to decline or even disappear from the market, causing the ultimate outputs to be redistributed across firms and industries (Yameogo et al., 2021). Then, the less polluting businesses with more resources can show a faster rate of progress, especially in the tertiary industry. As an alternative, the initiative may result in better-designed laws and stimulate new industries based on developing technological advances (Liu et al., 2021). That is why environmental information disclosure may lead to changes in resource reallocation among local businesses and industries that may encourage the improvement of regional industrial structure. Environmental regulations can significantly impact the financial performance of companies, investment decisions, and the spread of green technology innovation (Gu and Zheng, 2021), while also allowing them to decompose their production operations and utilize the country-specific advantages of countries outside their home territory. In countries with severe environmental rules, polluting businesses will relocate to countries with lax environmental regulations (Zhang M. et al., 2020). Researchers believe that environmental regulations play a significant role in screening the quality of foreign direct investment and restricting pollution-intensive enterprises to boost their green technology innovation capabilities (Pan and Chen, 2021). China’s government has prioritized enforcing appropriate environmental legislation to combat climate change and foster green technology innovation through FDI.

Recent years have seen a steady increase in scientific and technical resources in various parts of the world. To put it another way, from 1995 to 2017, the percentage of national research and experimental development financing to GDP climbed from 0.57 to 2.13%, and the intensity of that funding increased from 1.66 to 2.13% between 2009 and 2017. China’s technical level has remained stagnant despite an increase in investment in research and technology resources. According to Wang et al. (2022), China’s industry has a low level of innovation, indicating that the available scientific and technological resources have not been utilized. According to a number of studies, resource misallocation is a common problem in China’s economy (Zhao et al., 2022). According to several pieces of research, China’s economic growth can be boosted by increasing the efficiency of resource allocation efficiency (Fan et al., 2021). This has resulted in a growing interest in resource allocation in recent publications. Numerous studies have focused on China’s domestic market distortions and official interventions contributing to resource misallocation. In related research, it has been discovered that FDI value and pattern are essential in understanding how and why China has become one of the most important emerging economies in the world’s market (Wellalage et al., 2021). Against this backdrop of Chinese FDI contributing to the improvement of domestic FDI, this article examines whether and how different variables of Chinese FDI contribute to this improvement.

The article "Does industrial up-gradation, environment regulations, and resource allocation impact on foreign direct investment: Empirical evidence from China" was retracted in 2025. Reasons: an official misconduct investigation; compromised peer review; a compromised editor; unreliable results or conclusions.

This study aims to investigate the impact of industrial upgradation, environmental regulations, and resource allocation impact on foreign direct investment. As a result, the following research topic is the focus of this investigation. What effect will environmental regulation have on the performance of FDI in China as its economy grows? China’s FDI level will be examined to address the following concerns by analyzing the effects of environmental rules on China’s economic growth and population aging and their synergistic effects. Environmental regulations, industrial upgradation, environmental rules, and resource allocations in China have been extensively investigated in previous research. There are several examples of this, such as the national level (Ramzan et al., 2022), the city level (Soo et al., 2021), and the regional level (Ju et al., 2020). The impact of FDI on several economic indicators has also been examined by academics (Yang et al., 2020; Lv et al., 2021; Zhang, 2021). The synergistic effects of different environmental restrictions and two-way FDI on economic aspects have not been examined in any study. According to these findings, this article aims to fill the research gap with the following novelties. First, this study compares the various effects of environmental legislation on foreign direct investment. Second, we also looked into the impact of technological advancement on FDI. It is also crucial that this study takes the first step toward accounting for FDI resource allocation in policymaking. This study used empirical analysis to examine the impact of population aging and economic growth on FDI, considering socioeconomic and demographic aspects. The following are the study’s breakthroughs: A number of studies have looked at the impact of formal empirical estimators on FDI from 2005 to 2018 across China’s 30 provinces. The Dumitrescu–Hurlin (D-H) Panel causality test is used to evaluate the causal relationship between variables in this study.

The article "Does industrial up-gradation, environment regulations, and resource allocation impact on foreign direct investment: Empirical evidence from China" was retracted in 2025. Reasons: an official misconduct investigation; compromised peer review; a compromised editor; unreliable results or conclusions.

Here is the rest of the article’s logical structure: Relevant studies on science and technology resources are reviewed in Section “Literature review” of this document, including studies on the agglomeration degree of regional science and technology resources. Models, variables, and data sources are all covered in Section “Data and methods.” Scientific and technological resources are tested for spatial correlation in Section “Results and discussions.” Section “Conclusion and policy recommendations” focuses on empirical testing and analysis, including data from spatial measurements within and between regions.

## Literature review

Economic growth and environmental restrictions in China are increasing at an ever-increasing pace, and local governments in China’s provinces and cities will progressively be compelled to limit the entry of export corporates that are highly polluting and use a lot of energy. So that they can accomplish the desired effect of “decontamination and cleaning,” provinces and cities across China are abandoning their original development models in favor of more innovative ones that rely heavily on foreign investment (Fatai Adedoyin et al., 2021). With the help of eco-friendly foreign-funded firms, Chinese provinces and cities have accelerated national green innovation through the technology knock-on effects they generate (Tang et al., 2022). Foreign-funded Chinese companies benefit from the country’s increasingly strict environmental regulations, for example, investing in new devices and improving manufacturing capabilities (Wu and Lin, 2022). The increased prices of technology are supposed to lead to a long-term decline in international investment in financially advanced nations. Chinese local governments are also engaging in an environmental policy game to attract foreign investment (Zhang et al., 2021c). Therefore, local governments in China may play with each other to reduce environmental rules and values to acquire a competitive benefit in a strong market struggle, which fascinates foreign investment. The overall effect of environmental regulations in China has been to significantly impede foreign direct investment to achieve the overarching purpose of environmental rules, according to local governments in China.

To achieve industrial upgrading, short-term environmental rules will boost the marginal costs of corporates and have a cluttered effect on R&D expenditures (De Santis et al., 2021). Failure to achieve industrialization necessitates relocating foreign-funded firms to regions and countries with poorer environmental regulations, even though emission controls are costly (Zhang and Song, 2021). As for the “innovation compensation” effect (Ngo, 2022), companies are compelled to introduce cutting-edge technology and equipment, innovate technologically, and adjust product structure from a long-term perspective because of environmental regulations and rising marginal costs. Companies use the abovementioned strategies to absorb the high pollution costs, perform the necessary industrial modifications, and maintain their position as industry leaders (Wang and Zhang, 2020; Bekun, 2022). Another issue is that domestically funded firms with comparatively outdated manufacturing technologies will find it increasingly difficult to compete against foreign-funded firms with more advanced production capabilities in terms of global product demand and commodity export structure. Businesses in the United States will be negatively affected by this. With more advanced production technology, foreign-funded companies with more advanced production technology force domestic firms to upgrade their production technologies, indicating that the process of industrial upgrading has been completed (Zhang J. et al., 2020). Fourth, under stricter environmental rules, foreign-funded companies that have completed industrial upgrades are still lucrative and will spend further from a broader perspective. Ecological rules enormously boost FDI from the standpoint of industrial upgrading.

The article "Does industrial up-gradation, environment regulations, and resource allocation impact on foreign direct investment: Empirical evidence from China" was retracted in 2025. Reasons: an official misconduct investigation; compromised peer review; a compromised editor; unreliable results or conclusions.

Increasing environmental regulatory requirements will drive businesses to estimate their growing environmental expenses based on the effect of “following costs,” even if technology advancements remain constant. As a result of the aforementioned circumstances, businesses have seen their marginal costs soar, and their allocation of resources and production efficiency plummet (Kinyondo and Huggins, 2021). For this reason, foreign-funded businesses that have difficulty allocating their resources efficiently will be forced to seek other markets where environmental rules are less stringent as pollution control expenses rise. Instead, corporations will be encouraged to innovate and produce more due to appropriate environmental restrictions. Optimizing resource allocation will be encouraged to improve economic performance, so enterprises can incorporate pollution control expenses and maximize net profits (Qiu et al., 2021). Domestic firms with lower production technology levels face increased competition from foreign-funded firms with higher production technology levels, forcing domestic firms with higher production technology levels to optimize their resource allocation strategies. As a result, the industry has maintained a high manufacturing efficiency. It is possible for local businesses to improve their process efficiency by learning from smooth and technological international corporations, thus enhancing the city’s overall allocation of resources competence and green innovation through the new tech spillover effect (Huang and Lei, 2021). Finally, from a broader perspective, foreign-funded businesses nonetheless make significant profits under rigorous environmental rules by maximizing the allocation of resources and stimulating additional investment. Ecological restrictions have a substantial impact on foreign direct investment from a resource allocation perspective.

The article "Does industrial up-gradation, environment regulations, and resource allocation impact on foreign direct investment: Empirical evidence from China" was retracted in 2025. Reasons: an official misconduct investigation; compromised peer review; a compromised editor; unreliable results or conclusions.

As a result of the divergent views on resource distribution, current research has been divided into two categories: studies on resource distribution and those looking at resource maldistribution. The misallocation of resources is the subject of the first body of research. Mngumi et al. (2022) reviewed many studies and found that resource allocation efficiency is essential in explaining differences in total factor productivity (TFP) between countries. An effective reallocation of resources between businesses can enormously impact economic growth (Pellow et al., 2020; Peng, 2020; Liu et al., 2022). TFP dispersion, a measure popularized by Zhou et al. (2020), has been used extensively in research looking at firm-level misallocation. As a result, the importance of in-firm resource allocation has been disregarded to some extent. For macro-outcomes, including business cycle volatility, TFP, and economic growth, Yu and Li (2020) revealed that how resources are allocated inside a firm has a significant impact. Yu and Wang (2021) study endogenous product selection within firms and point out that resource allocation within firms may be more essential than resource allocation across companies, emphasizing the importance of resource allocation within firms. Factor misallocation in China is depicted by Wen and Zhang (2022) in the form of stylized facts. Although numerous studies have attempted to solve China’s resource misallocation problem, the majority have concentrated solely on internal issues, government engagement, and specific policies (Brandi et al., 2020; Wu et al., 2021; Qiu et al., 2022). There appear to be few studies that have explicitly examined the influence of China’s internationalization *via* FDI on the allocation of internal resources, especially at the micro-level.

The article "Does industrial up-gradation, environment regulations, and resource allocation impact on foreign direct investment: Empirical evidence from China" was retracted in 2025. Reasons: an official misconduct investigation; compromised peer review; a compromised editor; unreliable results or conclusions.

Foreign direct investment from emerging economies is the subject of the second strand of research in our article (EEs). A growing number of economic studies have recently focused on emerging economies as a source of FDI (Zhang et al., 2021b; Zhou et al., 2021; Wang and Zhang, 2022). Numerous researchers have conducted research on FDI trends and motivations, such as in previous studies (Cai et al., 2020; Khan and Chaudhry, 2021; Zhang et al., 2021b). Research on the influence of FDI on domestic performance has gotten less attention because of the paucity of FDI in firm-level data (Wei and Lihua, 2022). However, empirical evidence shows that enterprises’ participation in FDI is quite heterogeneous. Data collected at the firm level does aid in FDI research (Alola et al., 2022). There has been an increase in the use of business data in recent studies (Ngo, 2022). FDI patterns, in general, and Chinese enterprises in particular, matter to the performance of firms, according to the majority of the data (e.g., Wu et al., 2020; Shao et al., 2021; Xie et al., 2021). As a result, more information on enterprises’ FDI statistics is required to understand better how FDI affects resource allocation inside firms. We can discern the roles played by different types of FDI on firms’ resource allocation efficiency thanks to our unique information on the impact of Chinese enterprises’ outward foreign direct investment (OFDI) on internal resource allocation efficiency.

As a vital national resource, scientific and technological resources have recently gained scholarly attention. The effectiveness of scientific and technical resource allocation can be measured using various index systems and function models. China’s industrial R&D efficiency was determined to be low by Xiang et al. (2022), who used new product development as an output index, total R&D funding, and the number of technical staff as input indicators (Ahmad et al., 2021). To determine China’s high-tech industry’s innovation efficiency, Zhu and Xu used the stochastic frontier production function, which uses sales revenue from new products as a production predictor of R&D projects, R&D capital spending as an input predictor, and R&D employees as an indicator of input expenses. Gonzalez-Trevizo et al. (2021) found China’s industrial expenditure inefficient using the directional distance function. According to Dong et al. (2021), a generalized Cobb–Douglas production function was utilized to measure the company’s information capital by calculating the R&D accumulated capital. R&D initiatives like product and technology innovation have been demonstrated to boost the productivity of businesses. The efficient distribution of scientific and technological assets across cities is affected by a phenomenon known as spatial agglomeration, which Fan discovered using the exploratory spatial data analysis (ESDA) method. They developed an assessment index method to measure the distribution of regional scientific and technological resources, which they utilized to examine the variations in allocation of scientific and technical resources between regions by calculating Gini coefficients and Theil indexes. Data Envelopment Analysis (DEA) super-efficiency CCR model and Malmquist index model were used by Du et al. (2021) to analyze China the effectiveness of technology and science resource allocation using ESDA. They used the innovative input–output index system for this. They looked at the distribution of technology and science resources in different provinces based on their spatial agglomeration features. The data on “financial resources” and “innovative achievements” from 2009 to 2016 were used by Pan and Chen (2021) to develop an appropriate index system for evaluation. Regional disparities in China’s allocation of technology and science assets remain and are expanding rapidly, despite China’s increased capacity to allocate funds.

The article "Does industrial up-gradation, environment regulations, and resource allocation impact on foreign direct investment: Empirical evidence from China" was retracted in 2025. Reasons: an official misconduct investigation; compromised peer review; a compromised editor; unreliable results or conclusions.

A “government–various innovation entities in the region have established market” joint allocation model and cooperative development by distributing regional innovation, realizing redistribution, promoting technological and scientific development, and improving the operational efficiency of scientific and technical activities (Zhao et al., 2022). Xing and Kolstad (2002) claim that invention resources will not flow into businesses on their own under an open sharing method for scientific and technological resources and that businesses need to build a culture of support for sharing innovation resources. Yu and Wang (2021) developed a rational, cooperative innovation benefit distribution method based on basic game theory principles to ensure resource sharing based on the logic of collaborative innovation. China’s Yangtze River Economic Belt (YREB) is home to some of the world’s most technologically advanced regions. A recent survey shows that scientific and technical resources and collaborative innovation are more concentrated in these areas than elsewhere. Regional variations are fully evident in the gradient pattern of central, eastern, and western regions. However, while the Yangtze River Economic Belt as a whole has some synergistic innovation effects, the synergistic innovation effects among the center and western regions are pretty low. They feel that government funding should be more focused, scientific research should be better funded, and private enterprises and markets should be given more freedom to innovate (Duan et al., 2021). Heterogeneous research and development can not only be avoided, but it can also help address China’s technological innovation challenge.

The article "Does industrial up-gradation, environment regulations, and resource allocation impact on foreign direct investment: Empirical evidence from China" was retracted in 2025. Reasons: an official misconduct investigation; compromised peer review; a compromised editor; unreliable results or conclusions.

## Data and methods

### Theoretical explanations and model constructions

This article uses data from 30 Chinese provinces from 2005 to 2019 because of the data accessibility and dependability. Data utilized in this article all originate from the Chinese economy book of the year. According to Hsu et al. (2021), “upgrading industrial structure in an area” refers to transitioning from primary to tertiary industries. The shift expresses this change in industrial structure in the share of production value across different industries. Environmental restrictions may be strengthened due to the ecological information disclosure program. Companies in more transparent cities are subject to stricter regulations because of their ability to handle rebellious local governments and pollutants successfully. It is possible that environmental regulations could force polluting businesses to scale back their operations or even exit the market entirely. This shifts the output results among businesses and industries (Zhang and Qiu, 2022). As a result, the tertiary industry can demonstrate faster progress, particularly in light pollution. While this program may lead to better-designed rules and the creation of new initiatives from emerging technologies, it may also have the opposite effect (Luo et al., 2021). Consequently, we believe that environmental information disclosure could help improve the regional industrial structure, which could lead to changes in the allocation of resources among local businesses and industries. First, as China’s trade introduction continues to expand in depth, foreign direct investment is now one of the significant aspects of economic growth. Second, as the excessive expansion of foreign direct investment in the scale of resource-based companies proceeds, the problem of environmental degradation is becoming more and more concerning. Foreign direct investment in each region is converted into RMB using RMB’s yearly average exchange rate versus the USD (FDI). In addition, for the stability test, this article substitutes the actual use of foreign direct investment (Ye et al., 2021) with the percentage of GDP derived from FDI per area. Table 1 presents the description of each variable and data source.

**TABLE 1:** Variable description and data source.

Variables	Unit	Definition	Source
FDI	Yuan	Investment of enterprises with funds from foreign funding	Chinese trade foreign economics statistical yearbook
IU	The proportion of output value	The industrial structure of upgrading is assessed by the proportion of output value of the treasury	Chinese yearbook
ER	percentage	The proportion of total sewage in change GDP	Chinese yearbook
RA	100 RMB Yuan	Fix investment	Chinese yearbook
PA	65^+^ years	Percentage of the total population	Chinese yearbook
GDP	Yuan	GDP deflated based on the 2,000	Chinese yearbook

COIEC refers to the Chinese investment enterprise catalog of the ministry of commerce in China.

The article "Does industrial up-gradation, environment regulations, and resource allocation impact on foreign direct investment: Empirical evidence from China" was retracted in 2025. Reasons: an official misconduct investigation; compromised peer review; a compromised editor; unreliable results or conclusions.

Measurement methods for monitoring environmental regulation are currently broken down into cost and performance-based environmental regulation measures. The lack of government statistics on pollution costs and investments in environmental regulation may make it challenging to measure environmental regulation. A lower government standard for environmental pollution to entice foreign-funded businesses is closely linked to the gross industrial output value, which means that the cost of pollution control is often used as a yardstick for regulating the environment, which can lead to severe endogenous problems (Wu et al., 2020). The purpose of this research is to create a comprehensive environmental regulatory intensity index by making use of a linear weighted sum approach and the two separate indices of SO2 removal rate and industrial smoke dust removal rate in each region, given that cost-based environmental regulation indicators are lacking (Liu et al., 2021). Technology resources include RDE, TPE investment, and scientific and technological expertise (RDP). The two most common ways to measure technology capital investment are the R&D capital stock and the internal expenditure of R&D funds. Measurement of R&D capital stock is required to effectively quantify the impact of technological capital investment on regional innovation output. Using data from previous studies (Shuai and Fan, 2020), we may infer that this study’s urbanization rate is a key control variable. The urbanization rate is computed as the ratio of the population aging to the total population at the year’s end. A scatterplot of variables is given in Figure 1.

**FIGURE 1:** Scatterplot of variables.

Major problems may arise if panel data cross-sectional dependency (CD) is ignored (Dumitrescu and Hurlin, 2011). Therefore, three tests as CD test by Friedman (1937), Frees (1995), and Pesaran (2004) are employed to decide on a suitable panel technique, whereas an explanation of the mathematical form of the CD ratio test can be given as follows:


(1) $$C\,D=\sqrt{2\,T/N\,\left(N-1\right)}\,\left(\sum_{i=1}^{N-1}\sum_{j=i+1}^{N}\rho \,i\,j\right)\,N\,\left(0,1\right)$$

(2) FRI=(T-1)[2N∑i=1N-1∑j=i+1Nγij+1]χ(T-1)2

(3) $$F\,R\,E=\frac{\left(\text{T}-1\right)\,\,\left[\frac{2}{N}\,\sum_{i=1}^{N-1}\sum_{j=i+1}^{N}\gamma \,i\,j+\frac{1}{T}\right]}{S\,E\,\left(Q\right)}\,N\,\left(0,1\right)$$

In this context, the coefficient of residual affiliation in individual OLS regression is denoted by the letter ρ. The estimated value of ij denotes the rank coefficient of Spearman’s matrix, and the standard error of the Q distribution is denoted by SE (Q). The Fisher test is a first-generation unit root test that assumes Panel CD, and the formula for it can be written out as follows:


(4) Δy=i,tα+iγyi+i,t-1∑j=1kαjyi,t-1+εti,

where Δyi, t denotes the first difference of yi at the T at i-th observation of the panel, same as γ, εi, and t is the random disturbance term. Assuming the CD (Pesaran, 2007), CADF is used as the second generation unit root test and can be expressed as follows:


(5) $$\begin{array}{l} \Delta {\text{y}}_{\text{i},\text{ t }}=\alpha_{i}+\beta_{i}{}^{*}y_{i,t-\text{1}}+d_{0}y_{t-\text{1}}+\sum_{j=0}^{p}dj+1\Delta y_{i,t-j}\\ +\sum_{k=1}^{p}Ck\Delta y_{i,t-k}+\mu_{i,t} \end{array}$$

Cross-sectionally augmented Im-Pesaran-Shin (CIPS) can be measured by the mean of *t* statistics of the parameter β* in the CADF model.


(6) $$\mathrm{CIPS}=\sum_{i=1}^{N}\frac{t}{N}$$

Co-integration testing is the next step. There is a long-term correlation between the concern variables when both series are integrated in the same order. Co-integration can be used to spot long-term equilibrium processes. Durbin Hausman’s group men co-integration test has been used in this procedure (Westerlund and Edgerton, 2007). The CD ratio can be used in this test, and prior knowledge of the integration sequence of variables is not required. As a result, it can be put to use in the following scenarios.

The article "Does industrial up-gradation, environment regulations, and resource allocation impact on foreign direct investment: Empirical evidence from China" was retracted in 2025. Reasons: an official misconduct investigation; compromised peer review; a compromised editor; unreliable results or conclusions.

### Augmented mean group and long-term relationship

When models have heteroscedasticity, CD, and serial correlation, panel estimators can lead to inferior and even inconsistent estimates that are deceptive, as detailed common correlated effects (CCEs) were established by Chudik and Pesaran (2013) to overcome these issues. Compared to first-generation econometric approaches, this approach has significant advantages. No consideration is given to estimating unobserved common variables and loading variables. The Augmented Mean Group (AMG) algorithm developed by Bond and Eberhardt (2013) will be used in this investigation. AMG can handle non-stationary variables in the approximation of parameters without restriction, as can be seen in the main panel model shown below:


(7) $$l\,n\,F\,D\,I_{i\,t}=\beta \,0+\beta \,1\,l\,n\,I\,U_{i\,t}+\beta \,2\,l\,n\,E\,R_{i\,t}+\beta \,3\,l\,n\,R\,A_{i\,t}+\beta \,4\,l\,n\,P\,A_{i\,t}+\beta \,5\,l\,n\,G\,D\,P_{i\,t}+\varepsilon_{i\,t}$$

The first differenced form and the T-1 period dummy are used to measure the aforementioned equation (M).


$$\Delta \,F\,D\,I_{i\,t}=\beta \,0+\beta \,1\,l\,n\,I\,U_{i\,t}+\beta \,2\,l\,n\,E\,R_{i\,t}+\beta \,3\,l\,n\,R\,A_{i\,t}+\beta \,4\,l\,n\,P\,A_{i\,t}$$

(8) $$+\beta \,4\,l\,n\,G\,D\,P_{i\,t}+\sum_{t=2}^{T}p\,t\,\left(A\,D\,t\right)+\mu_{i\,t}$$

Dummies for period dummies can be found in ADt, which denotes the first difference between T-1 period dummies. Pt variables are substituted with T variables in the next step, which signifies the dynamic technique.


$$\Delta \,F\,D\,I_{i\,t}=\beta \,0+\beta \,1\,l\,n\,I\,U_{i\,t}+\beta \,2\,l\,n\,E\,R_{i\,t}+\beta \,3\,l\,n\,R\,A_{i\,t}+\beta \,4\,l\,n\,P\,A_{i\,t}$$

(9) $$+\beta \,4\,l\,n\,G\,D\,P_{i\,t}+d\,1\,\left(\delta \,t\right)+\mu_{i\,t}$$

(10) $$\Delta \,F\,D\,I_{i\,t}-\delta \,t=\beta \,0+\beta_{1}\,l\,n\,I\,U_{i\,t}+\beta_{2}\,l\,n\,E\,R_{i\,t}+\beta_{3}\,l\,n\,R\,A_{i\,t}+\beta_{4}\,l\,n\,P\,A_{i\,t}+\beta_{4}\,l\,n\,G\,D\,P\,i+\mu_{i\,t}$$

In addition, this study used the common correlated effects mean groups (CCE-MG) estimator for its robustness.

### Dumitrescu–Hurlin panel causality test

Heterogeneous panel data can be tested using this technology. In addition to considering the CD ratio, this methodology implies that the time dimension and the cross-sectional area are related. Unbalanced data can generate beneficial results (Dumitrescu and Hurlin, 2012). The causality of a panel can be expressed as follows:


(11) Y=i,tαit+∑k=1kγ(k)y+i,t-k∑k=1kβi(k)x+i,t-kεit

This equation displays β1 + β2 + β3 + … + βk, where αi represents each unique fixed effect, lag parameters are represented by γ(k), the lag length K, and the slope of the parameters is represented by βi(k). Here is what the D-H panel test’s hypothesis is:

Null hypothesis; H0: βi = 0 (homogenous results of causality).

Alternative hypothesis; H1: βi ≠ 0 (heterogeneous results of causality).

Because the panel data do not show any correlation between cause and effect, the null hypothesis cannot be accepted or rejected based on its probability values alone. The following is an explanation of this approach:


(12) W=N,THnc1N∑i=1NWi,t

## Results and discussion

Table 2 shows the descriptive statistics for each variable and shows that no problem can create a problem for the empirical estimation.

**TABLE 2:** Descriptive statistics.

Variable	Mean	Std. deviation	Minimum	Maximum
LFDI	7.885	0.214	0.674	10.771
LIU	5.228	0.679	0.877	8.659
LER	8.354	0.238	0.547	11.554
LRA	9.986	0.562	0.655	10.986
LPA	4.875	0.234	0.471	9.489
GDP	6.558	0.428	0.675	10.326

Likewise, Table 3 presents the result of pairwise correlation. Similarly, industrial upgradation positively correlates with FDI at a 1% significance level. Environmental regulations are inversely associated with the explained variable at a 1% significance level. Similarly, resource allocation, population aging, and economic growth are positively associated with the explained variable.

The article "Does industrial up-gradation, environment regulations, and resource allocation impact on foreign direct investment: Empirical evidence from China" was retracted in 2025. Reasons: an official misconduct investigation; compromised peer review; a compromised editor; unreliable results or conclusions.

**TABLE 3:** Pairwise correlation test.

	LFDI	LIU	LER	LRA	LPA	GDP
LFDI	1					
LIU	0.694	1				
LER	–0.324	0.258	1			
LRA	0.452	0.369	0.661	1		
LPA	0.657	–0.654	0.489	0.702	1	
GDP	0.734	0.398	0.563	0.591	0.692	1

### Cross-sectional dependency test and cross-sectionally augmented Im-Pesaran-Shin unit root test

For empirical research using panel data, the cross-sectional dependence (CSD) issue is likely to be a concern, as well as homogeneity and serial correlation. This work employs advanced panel data econometric methodologies to manage endogeneity, CSD, and serial correlation to address the aforementioned issue. Table 4 shows the findings of the CD test, which is the first step in determining whether or not a patient has CSD. CSD is a statistically significant factor in this study’s results. As a result, shocks in one nation may impact data from other countries included in the study. To determine which regression estimation method is best suited for the data, the series must be verified for stationarity. The CIPS unit root test (Pesaran, 2007) and other panel data analysis unit root tests have lately gained traction in the literature. Table 4’s CIPS results are shown at the bottom of the table. If the series is not stationary, then the null hypothesis is that the series has a unit root. Because all factors have unit roots at the level, the sequence is initially integrated into the first order, transforming to stationary performance after the first variation.

**TABLE 4:** CSD and CIPS unit root test.

Selected model	Pearson (CD)	Frees (Q)		Friedman (CD)
Statistics	32.912*	6.899*		265.41*

**CIPS unit root test**				

**Variable**	**Level**		**First difference**	

LIU	−2.223**		−4.558	
LER	−1.045		−5.899*	
LRA	−2.012		−4.524*	
LFDI	−3.966*		−7.569	
LPA	−2.999**		−3.875	
LGDP	−3.387*		−4.623	

*, ** means 1% and 5% significance level.

To determine whether the selected variables have a long-term relationship, it is necessary to conduct the co-integration test and this study uses the co-integration test proposed by Westerlund and Edgerton (2007). An essential aspect of this study’s usage of the test is its ability to accommodate variation in both long-term co-integration and short-term dynamics (Westerlund and Edgerton, 2007). In addition, it is appropriate for cross-sectional dependency. The bootstrap settings for many repetitions of the co-integration test are also available in this study’s bootstrap test. The Gt and Ga (group mean test) were suggested by Westerlund and Edgerton (2007) to investigate the hypothesis that at least one of the units is co-integrated. Table 5 demonstrates that the Gt, Ga, Pt, and Pa test statistics are all significant according to the Westerlund test. However, according to the given outcome, this study rejects the null hypothesis H_0_ of no co-integration among the selected variables, but the obtained results insist us to accept the alternative hypothesis of co-integration among the variables. On behalf of outcomes, this study can proceed further to long-run estimators.

The article "Does industrial up-gradation, environment regulations, and resource allocation impact on foreign direct investment: Empirical evidence from China" was retracted in 2025. Reasons: an official misconduct investigation; compromised peer review; a compromised editor; unreliable results or conclusions.

**TABLE 5:** Westerlund co-integration test.

Statistics	Value	*Z*-value	*P*-value	Robust *P*-value
G_t_	−4.285	6.745	1.000	0.000
G_a_	−2.996	4.852	1.000	0.225
P_t_	−7.489	9.887	1.000	0.005
P_a_	−1.510	7.392	1.000	0.633

### Long-run outcomes of augmented mean group and common correlated effects mean groups estimators

According to this study, industrial upgrading, environmental laws, resource allocations, population aging, and economic growth impact foreign direct investment in Table 6. According to the coefficient, FDI is favorably connected with LIU’s industrial structure. According to the AMG and CCE-MG estimators, a 1% rise in this component would lead to a 0.452 and 0.488% increase in foreign direct investment, respectively. This connection is rationally explicable. The immediate effect of technological innovation on industrial structure upgrades was favorable, but outside of the region, it had a suppressing influence on industrial structure upgrades. To put it another way, this indicates that technological innovation has a favorable impact on sectors and goods, as well as a direct effect on the conventional level of innovation and a breakthrough in technology. Businesses will gain a long-term competitive edge by gradually phasing out obsolete technology industries, which will have a direct impact. Technology spillover significantly impacts the surrounding area, as does the local population’s absorption and use of that technology. Therefore, the effect was detrimental, although none of the impacts were statistically significant. As a result, technical advancement in one sector may harm industrial structure upgrades elsewhere; however, this effect is difficult to detect. This is in line with most academics’ findings (Qiu and Wu, 2010; Xin, 2014; Gong et al., 2015). Scholars, on the contrary, have come to differing views. For instance, Zhu (2007) quantified China’s industrial structure’s coordination and linkage. Researchers found that China now has a low level of technological innovation and an unbalanced structure in its industrial sector. During coordinated development, the educational level was low, and the industrial structure was relatively simple, resulting in a cause-and-effect relationship. Overall, Wang and Wei (2018) found that from 1995 to 2015, China’s technological innovation capabilities and industrial structure optimization and upgrading were continuously increasing, especially since the beginning of this century. Even though there was an increase in coupling coordination, the total level of coordination and coupling remained low. This supports the findings of this research, which show that technological innovation has considerably aided in restructuring the industrial structure in recent years.

The article "Does industrial up-gradation, environment regulations, and resource allocation impact on foreign direct investment: Empirical evidence from China" was retracted in 2025. Reasons: an official misconduct investigation; compromised peer review; a compromised editor; unreliable results or conclusions.

**TABLE 6:** Long-run outcomes of **augmented mean group** (AMG) and CCE-MG estimators.

	AMG estimator		CCEMG estimator	
	Coefficient	Std. error	Coefficient	Std. error
LIU	0.4522*	0.3269	0.4987*	0.2913
LER	−0.6952*	0.1378	−0.7379*	0.1937
LRA	1.6541*	0.5674	0.9963*	0.3356
LPA	−0.2396**	0.0992	−0.3198**	0.1201
LGDP	0.9623*	0.2911	0.8755*	0.3574
Cons.	−0.7264*	0.2938	−0.6329*	0.2254

*, ** means 1% and 5% significance level.

Furthermore, environmental regulations could be a factor that affects the amount of FDI inflows. If this factor was to rise by 1%, FDI inflows would fall by 0.695 and 0.737%, respectively, using the approaches described. Environmental rules have been developed due to growing concern, but their effectiveness is limited without FDI coordination in their implementation. Therefore, there is clear evidence that RE affects FDI, as shown by the significant negative direct ER coefficients at the 1% significance level. According to AMG and CCEMG models, the “Porter hypothesis” exists in China when the AMG and CCEMG models are used for empirical analysis, indicating that ER impacts FDI. The pollution haven hypothesis holds that countries with lax environmental regulations are more likely to attract FDI as a result of the formation of pollution havens. Most publications examine the RTB effect in less developed nations (Liu et al., 2020; Ngo, 2022). Many additional studies, such as Hu D. et al. (2021), focus on the multi-national corporations’ decision to invest in more or less regulated nations, depending on corporate social responsibility or other variables regarded as more significant.

Foreign direct investment positively correlates with allocating scientific and technical resources. Foreign direct investment would climb by 1.654 and 0.996%, respectively, if this factor increased by 1%. This figure depicts the flow of scientific and technical assets between areas. This has a significant impact on regional innovation production. Interregional movements of technological capital and personnel have extended the economic scope of each technology in each region. Regional economic integration has also been boosted by an increase in the transfer of scientific and technological resources across regions. As knowledge and technology spread and economies integrate, scale returns will significantly impact innovation production across regions and nations. Furthermore, the impact of regional innovation production on the movement of scientific and technical team members is more significant than the impact of regional innovation output on the mobility of technological unit capital. A key factor in increasing regional innovation output is removing obstacles that prevent the free flow of scientists and technologists and fully appreciating the resource redeployment that results from their presence. To make matters more complicated, regression analysis shows that each invention in the scientific and technology resource sector has similar allocation policies. The calculated coefficients for each variable have a consistent sign and level of significance, demonstrating the robustness of the estimates in this work. The coefficient shows that the movement of scientists and technologists between colleges and institutions in different provinces can greatly increase regional FDI inflows after considering inter-regional data.

The article "Does industrial up-gradation, environment regulations, and resource allocation impact on foreign direct investment: Empirical evidence from China" was retracted in 2025. Reasons: an official misconduct investigation; compromised peer review; a compromised editor; unreliable results or conclusions.

Foreign direct investment inflows are also declining due to the aging population. According to the AMG and CCE-MG estimates, a 1% increase in this component would reduce FDI inflows by 0.239 and 0.319%, respectively. FDI development is hampered by the presence of PA, which indicates that an increase in PA will impede FDI into provinces. For example, it may be because of pollution-based investments. The “pollution refuge” effect is stronger than the “pollution halo,” leading to environmental conditions decline, compounded by China’s aging population. Environmental rules slow FDI growth significantly, even if the aging population is a contributing factor. As a result, to accomplish ecologically sustainable, effective, and long-term growth in China, China must improve the transmission and administration of FDI, raise the threshold for international investment, and bring cleaner FDI with advanced tech and reduced energy consumption and low pollution.

Foreign direct investment is positively associated with GDP, which means that a 1% increase in GDP will increase the amount of FDI by 0.962 and 0.875% points, respectively. FDI and GDP have been linked, as shown in the research, which has significantly driven FDI into the country. The GDP is essential as a source of capital and boosts the economy’s competitiveness. China’s GDP results have been highly positive. Foreign investors consistently consider China one of the world’s best investment places. According to the regression model results, Chakraborty et al. (2015) have revealed similar results using FDI and GDP data from 1987 to 2011. However, their findings suggest that GDP and FDI are indeed linked. Our results could be contradictory because our data span from 1995 to 2015 when there has been a near-massive growth in international investors’ interest in Bangladesh since 2013. Bangladesh appears to be China’s choice for garment, footwear, and agro-industry investment.

The article "Does industrial up-gradation, environment regulations, and resource allocation impact on foreign direct investment: Empirical evidence from China" was retracted in 2025. Reasons: an official misconduct investigation; compromised peer review; a compromised editor; unreliable results or conclusions.

### Dumitrescu–Hurlin panel causality test

The D-H panel causality results in Table 7 disclose the relationship among variables. According to the given outcome, there found a bi-directional association between industrial upgradation and foreign direct investment, which infers that any significant variation in industrial upgradation would cause to change in foreign direct investment and vice versa. Similarly, the one-way causal association between foreign direct investment and environmental regulations explains that the policies related to both factors are not interconnected. Therefore, any significant change in environmental regulation would cause a change in FDI, and the feedback hypothesis does not exist. Similarly, there found the bi-directional causality between resource allocation and FDI and implies that any fluctuation in resource allocation would cause to change in the level of FDI. The same phenomenon will repeat for resource allocation. Moreover, there found a one-way causal association between population aging and foreign direct investment. Similarly, the feedback hypothesis was found between the GDP and FDI across the selected panel.

**TABLE 7:** Results of D-H panel causality test.

Null hypothesis	W-stat.	Prob.
LIU >> LFDI	7.9658	0.000
LFDI >> LIU	6.4558	0.001
LER >> LFDI	6.8951	0.000
LFDI >> LER	2.3485	0.666
LRA >> LFDI	9.7851	0.002
LFDI >> LRA	5.6598	0.000
LPA >> LFDI	3.5631	0.089
LFDI >> LPA	5.7469	0.000
LGDP >> LFDI	6.2356	0.000
LFDI >> LGDP	4.5487	0.000

## Conclusion and policy recommendations

Because of China’s recent economic boom and increased influx of technological and scientific resources, the country’s science and technology sector has risen fast. FDI is influenced by the allocation of scientific and technological resources, and we need to be more aware of this. Similarly, this research examines the effect of foreign direct investment on industry structure, environmental restrictions, population aging, and economic growth. This study uses the panel data of 30 provinces in China from 2005 to 2018 to structure a model, which includes both the technological allocation of scientific and technical resources and the utilization of spatial data analysis models to empirically analyze the different impacts of specified factors on foreign direct investment. The data for these provinces were collected using panel analysis. The empirical results show that industrial upgradation, resource allocations, population aging, and economic growth positively contribute to FDI inflows. Similarly, environmental regulations and population aging cause a decline in foreign direct investment. Moreover, this study uses the D-H panel causality test to investigate the causal association among selected variables.

The article "Does industrial up-gradation, environment regulations, and resource allocation impact on foreign direct investment: Empirical evidence from China" was retracted in 2025. Reasons: an official misconduct investigation; compromised peer review; a compromised editor; unreliable results or conclusions.

### Policy recommendations

The findings of this study have some fascinating policy implications for China’s foreign investment.

1. The local government environmental governance has a better chance of succeeding because of environmental decentralization, which encourages “top-to-top competition.” It is more likely that “one-size-fits-all approach” environmental governance measures will develop if local government competition severely lowers foreign direct investment.
2. Environmental control measures must be implemented to deal with foreign-funded firms’ pollution levels and development levels. In addition, the local authority competition mode in the framework of environmental decentralization must be further improved. This environmental information disclosure program must be improved to boost industrial structure upgrading in China’s regions.
3. Environmental regulations of all kinds should be improved in design and public participation promoted. As a result, more environmental information disclosure programs must be formed and improved in the long term to enable various stakeholder groups to enhance industrial development, particularly for the tertiary industry.
4. Investment in fixed assets and human capital will also affect the improvement of the regional industrial structure, and increased R&D spending and investment may have a favorable impact. It is, therefore, necessary to include all entities with a stake in upgradation to make the most use of available labor and cash.
5. Developing countries should take steps to make attracting FDI easier, such as reforming their external sectors, liberalizing financial flows, and bolstering their skills in R&D. Foreign direct investment has a positive effect on Chinese domestic investment, but this suggests that the lack of investment attractiveness and business climate of emerging countries compared to other countries may be caused by lower production costs and a higher rate of return due to the availability of cheap labor and other resources. Consequently, we can propose that China’s national development policy focuses on the productive exploitation of both domestic and foreign capital and the effective transfer of growth advantages into the development process.

The article "Does industrial up-gradation, environment regulations, and resource allocation impact on foreign direct investment: Empirical evidence from China" was retracted in 2025. Reasons: an official misconduct investigation; compromised peer review; a compromised editor; unreliable results or conclusions.

## Data availability statement

The original contributions presented in this study are included in the article/supplementary material, further inquiries can be directed to the corresponding author.

## Author contributions

JX: conceptualization, data curation, methodology, and writing—original draft. LC: data curation, visualization, supervision, writing—review and editing, and software. Both authors contributed equally to the article and approved the submitted version.
